# Authenticity Assessment of (E)-Cinnamic Acid, Vanillin, and Benzoic Acid from Sumatra Benzoin Balsam by Gas Chromatography Combustion/Pyrolysis Isotope Ratio Mass Spectrometry

**DOI:** 10.1155/2022/1747053

**Published:** 2022-09-07

**Authors:** Deshou Mao, Liu Hong, Lei Fu, Zhiyu Li, Jianhua Chen, Chengming Zhang, Yiqin Wu, Wen Xiong, Jin Wang

**Affiliations:** Technology Center of China Tobacco Yunnan Industrial Co. Ltd., Kunming 650231, China

## Abstract

Authenticity assessment of (*E*)-cinnamic acid, vanillin, and benzoic acid from various origins (*n* = 26) was performed using gas chromatography-isotope ratio mass spectrometry coupled with combustion and pyrolysis mode (GC-C/P-IRMS). For that reason, the above three compounds (1–3) from synthetic, natural, and Sumatra benzoin balsam (laboratory prepared, adulterated, and commercial) were investigated. The *δ*^13^C_V-PDB_ and *δ*^2^H_V-SMOW_ values for compounds 1–3 from synthetic samples (S1–S5) ranging from −26.9 to −31.1‰ and 42 to 83‰, respectively, were clearly different from those of authentic samples (N1–N4, L1–L9) varying from −29.8 to −41.6‰ and −19 to −156‰. In adulteration verification testing, for compounds 1 and 3, both *δ*^13^C_V-PDB_ and *δ*^2^H_V-SMOW_ data of A1 (5.0% added) and A2 (2.5% added) except A3 (0.5% added) fell into the synthetic region, whereas for compound 2, the *δ*^2^H_V-SMOW_ data of adulterated samples (A1–A3) fell into the synthetic region, and even the lowest adulterated sample A3 is no exception. With this conclusion, some commercial Sumatra benzoin balsam samples were identified to be adulterated with synthetic 1 (C1, C3, and C5) and synthetic 2 (C3, C4, and C5) but not with synthetic 3. GC-C/P-IRMS allowed clear-cut differentiation of the synthetic and natural origin of 1, 2, and 3 and definite identification of whether a Sumatra benzoin balsam was adulterated or not.

## 1. Introduction

Sumatra benzoin is a natural balsamic resin, exuded from a small tree, *Styrax benzoin* Dryander, grown extensively in Sumatra and Malaya, mostly cultivated in Vietnam, Thailand, and China [1]. Sumatra benzoin balsam was obtained by extraction, filtration, and vacuum distillation of the crude benzoin. It has a sweet, balsamic-cinnamic characteristic odor, which is used extensively as fixative in perfumery, food, and tobacco flavoring [2]. Driven by business interests, Sumatra benzoin balsam was often adulterated with synthetic flavors (*E*)-cinnamic acid (1), vanillin (2), and benzoic acid (3) (Figure 1) to claim that it was a better grade or “originated from Siam Benzoin” [3].

Current research on benzoin resin and balsam mainly focuses on the analysis of the different volatile and non-volatile components in various species or different places of origin [4–8], and little information is available about authenticity assessment. Concerning flavor authenticity and traceability, IRMS has been widely used due to the high precision of the method, the requirement for small samples, and the fact that the same technique can be used for almost any type of food or beverage [9–13]. Fink et al. studied hydrogen isotope ratio and carbon isotope ratio of the natural, synthetic, and semi-synthetic methyl cinnamate and showed that different sources of methyl cinnamate, ^2^H/^1^H and ^13^C/^12^C, have different distribution ranges [8]. This result shows that isotope analysis can be used to verify the authenticity of flavor compounds. In this study, we undertook the authenticity study of (*E*)-cinnamic acid (1), vanillin (2), and benzoic acid (3) from synthetic, natural, and Sumatra benzoin balsam through ^13^C/^12^C and ^2^H/^1^H isotope ratios measured by GC-C/P-IRMS analysis.

## 2. Materials and Method

### 2.1. Materials and Reagents

Synthetic (S1–S5) and natural (N1–N4) (*E*)-cinnamic acid, vanillin, and benzoic acid reference samples were purchased from Sigma-Aldrich, Tansoole, and J&K. Sumatra benzoin samples of four regions (Sumatra, Indonesia; Guangxi, China; Yunnan, China; Anhui, China) for laboratory prepared balsam (L1–L9) were available from Alibaba Group (Hangzhou, China). Commercial Sumatra benzoin balsam samples (C1–C5) were purchased from flavor companies including Biolandes, Mane, Apple, Boton, and Huabao. Other chemicals were purchased from Sigma-Aldrich. Solvents were redistilled before use.

### 2.2. Sample Preparation

Synthetic and natural reference samples were dissolved (2 mg/mL) in methanol, and the solutions were directly analyzed by GC-C/P-IRMS. After water washing, crushing, microwave-assisted extracting (0.5 h, 2.0 fold ethyl acetate as solvent), filtrating, and vacuum concentrating, the Sumatra benzoin samples were prepared into Sumatra benzoin balsam (yield 53%–72%, L1–L9), which were subjected to diluting to 10% solutions (*w/w*) using methanol followed by direct isotope ratio analysis. Adulterated Sumatra benzoin balsam samples (A1–A3) were designed by adding 5.0%, 2.5%, and 0.5% (*w/w)* corresponding synthetic reference (S1), respectively, to the above laboratory prepared balsams (L1). Likewise, all commercial and adulterated Sumatra benzoin balsam samples (C1–C5, A1–A3) were subjected to the same sample pretreatment before instrumental analysis.

### 2.3. GC-C/P-IRMS Conditions

A Finnigan Delta V Advantage isotope ratio mass spectrometer coupled to an HP 6890°N gas chromatograph via the open-splitof combustion and pyrolysis interface was used. The GC was equipped with an HP-INNOWAX fused silica capillary column (30 m × 0.32 mm × 0.25 *μ*m). The following conditions were employed: for GC: 1-*μ*L solution was injected in splitless mode (250°C); the injector temperature was 250°C; the initial oven temperature was 60°C, held for 1 min, then heated to at a rate of 180°C at 8°C/min, raised to 240°C at a rate of 6°C/min and held at 240°C for 17 min; the carrier gas was He at a flow rate of 1.5 mL/min. For ^13^C/^12^C: the solutions flow was online combusted into to CO_2_ at 960°C in the oxidative reactor (Al_2_O_3_, 0.5 mm×1.5 mm×320 mm) with Cu, Ni, and Pt (each 240 mm×0.125 mm); the water separated by Nafion membrane. For 2H/1H: the effluent from the GC were directed to a high-temperature ceramic tube (Al_2_O_3_, 0.5 mm×320 mm) and pyrolyzed to H_2_ at 1440°C. In addition, coupling GC isolink elemental analyzer system to the IRMS was realized for offline control determination of reference samples. Daily system stability checks were performed by measuring reference samples with known ^13^C/^12^C and ^2^H/^1^H ratios. The reference samples were using International Atomic Energy Agency (IAEA, Vienna, Austria) standards, and IAEA-601 used for ^13^C/^12^C and IAEA-601, and VSMOW used for ^2^H/^1^H, respectively. The isotope ratios are expressed in per mil (‰) deviation relative to the V-PDB and VSMOW international standards, and the calculation method is the same as reference [8]. In general, 6-fold determinations were carried out and standard deviations were calculated. The latter were ±0.2 and ±5‰ for *δ*^13^C_V-PDB_ and *δ*^2^H_V-SMOW_ determinations, respectively.

## 3. Results and Discussion

To check potential isotope discrimination in the course of sample preparation, the three synthetic reference samples under study (S1, 1–3) were subjected to the steps used for the laboratory prepared balsam. The data summarized in Table 1 showed that sample preparation did not affect the isotope values. The data from treated samples S1a did not differ significantly from those the untreated reference samples S1. The *δ*^13^C_V-PDB_ and *δ*^2^H_V-SMOW_ values of (*E*)-cinnamic acid (1), vanillin (2), and benzoic acid (3) from various origins (*n* = 26), including synthetic (*n* = 5), natural (*n* = 4), and Sumatra benzoin balsam (*n* = 9, laboratory prepared; *n* = 5, commercial; *n* = 3, adulterated with synthetic reference), are summarized in Table 2.

### 3.1. (E)-Cinnamic Acid (1)

In Figure 2, the ^13^C/^12^C and ^2^H/^1^H ratios determined for 1 in various samples are graphically correlated. Synthetic references (S1–S5, *n* = 5) showed *δ*^13^C_V-PDB_ and *δ*^2^H_V-SMOW_ data ranging from −26.9 to −27.6‰ and from −23.3 to −41.5‰. The *δ*^13^C_V-PDB_ and *δ*^2^H_V-SMOW_ values of natural references (N1–N4, *n* = 4), ranging from −29.8 to −30.7‰ and from −63 to −84‰, respectively, clearly differed from that of synthetic references. Laboratory prepared Sumatra benzoin balsams (L1–L9, *n* = 9) gave almost the same IRMS data like those found for 1 from natural references, ranging from −29.9 to −31.5‰ and from −56 to −103‰ of *δ*^13^C_V-PDB_ and *δ*^2^H_V-SMOW_ values, respectively. The *δ*^13^C_V-PDB_ and *δ*^2^H_V-SMOW_data of adulterated Sumatra benzoin balsams (A1–A3, *n* = 3), which added 5%, 2.5%, 0.5% synthetic (*E*)-cinnamic acid S1 to laboratory prepared balsam L1, respectively, ranged from −28.3 to −30.2‰ and from −37 to −61‰. Both *δ*^13^C_V-PDB_ and *δ*^2^H_V-SMOW_ data of A1 and A2 adulterated samples (except A3) almost fell into synthetic region compared with authentic samples (N1–N4 and L1–L9, *n* = 13), which further confirmed the former conclusion. With this conclusion, three commercial samples (C1, C3, and C5) were clearly identified to be adulterated with synthetic (*E*)-cinnamic acid.

### 3.2. Vanillin (2)

The correlation of *δ*^13^C_V-PDB_ and *δ*^2^H_V-SMOW_ data of 2 from the various origins is outlined in Figure 3. The graph shows distinct differences between synthetic (S1–S5, *n* = 5; *δ*^13^C_V-PDB_ from −27.8 to −29.0‰ and *δ*^2^H_V-SMOW_ from 42 to 83‰) and natural samples (N1–N4, *n* = 4; *δ*^13^C_V-PDB_ from −29.9 to −30.6‰ and *δ*^2^H_V-SMOW_ from −28 to −69‰). Compound 2 from laboratory prepared balsams (L1–L9, *n* = 9) exhibited *δ*^13^C_V-PDB_ and *δ*^2^H_V-SMOW_ values ranging from −29.8 to −31.4‰ and −19 to −82‰, respectively.

These data were in good agreement with those determined for 2 from natural samples (*n* = 4) (Figure 3). After adding 5%, 2.5%, and 0.5% synthetic vanillin S1 to laboratory prepared balsam L1, the *δ*^13^C_V-PDB_ and *δ*^2^H_V-SMOW_ values of adulterated Sumatra benzoin balsams (A1–A3, *n* = 3) ranged remarkably from −24.7 to −29.6‰ and from 58 to 13‰. The *δ*^2^H_V-SMOW_ data of adulterated samples (A1–A3, *n* = 3) fell into synthetic region compared with authentic sample (N1–N4 and L1–L9, *n* = 13), and even the lowest vanillin-adulterated sample A3 is no exception. Likewise, commercial sample C5 was definitely identified to be “significantly vanillin-adulterated,” while C4 and C3 were tenderly identified as “slightly vanillin-adulterated,” and commercial samples C1 and C2 were not adulterated.

### 3.3. Benzoic Acid (3)

The correlation of *δ*^13^C_V-PDB_ and *δ*^2^H_V-SMOW_ data of 3 from different origins is displayed in Figure 4. *δ*^13^C_V-PDB_ data for 3 from synthetic (S1–S5, *n* = 5) ranged from −28.7 to −31.1‰, and the *δ*^2^H_V-SMOW_ data varied from 34 to 70‰, whereas the data from natural (N1–N4, *n* = 4) were quite different (*δ*^13^C_V-PDB_ values from −37.7 to −41.6‰ and *δ*^2^H_V-SMOW_ values from −105 to −145‰). Compound 3 from laboratory prepared balsams (L1–L9, *n* = 9) exhibited ^13^C_V-PDB_ and *δ*^2^H_V-SMOW_ values ranging from −35.9 to −39.5‰ and −64 to −156‰, respectively, which were in good agreement with those determined for 3 from natural samples (*n* = 4) (Figure 4). The same isotope ratio changes of adulterated Sumatra benzoin balsams (A1–A3, *n* = 3; different amount of synthetic benzoic acid S1 added to L1) were observed as compound 1, varying from −29.3 to −36.3‰ and from −29.3 to −36.3‰ for *δ*^13^C_V-PDB_ and *δ*^2^H_V-SMOW_ values, respectively. Both the ^13^C/^12^C and ^2^H/^1^H ratio data of A1 and A2 adulterated samples (except A3) completely fell into synthetic region compared with authentic samples (L1–L9 and N1–N4, *n* = 13). Similarly, five commercial samples (C1–C5) were identified to be not adulterated with synthetic benzoic acid.

## 4. Conclusion

In conclusion, the *δ*^13^C_V-PDB_ and *δ*^2^H_V-SMOW_ values for authenticity assessment of (*E*)-cinnamic acid (1), vanillin (2), and benzoic acid (3) from various origins including synthetic, natural, and Sumatra benzoin balsam (laboratory prepared, commercial, and adulterated) were demonstrated. Despite the limited number of samples, GC-C/P-IRMS allowed clear-cut analytical differentiation of the synthetic and natural origin of 1, 2, and 3 and definite identification of whether a Sumatra benzoin balsam was adulterated or not. Future work will be done to extend the amounts of 1, 2, and 3 from natural plant sources, particularly Siam benzoin, which has antioxidative effect, economic value, and flavoring application [2], until finally build the IRMS database for their authenticity identification.

## Figures and Tables

**Figure 1:** Chemical structure of (1) (E)-cinnamic acid, (2) vanillin, and (3) benzoic acid.

**Figure 2:** *δ* ^13^C_V-PDB_ and *δ*^2^H_V-SMOW_ values of (E)-cinnamic acid from various origins.

**Figure 3:** *δ* ^13^C_V-PDB_ and *δ*^2^H_V-SMOW_ values of vanillin from various origins.

**Figure 4:** *δ* ^13^C_V-PDB_ and *δ*^2^H_V-SMOW_ values of benzoic acid from various origins.

**Table 1:** *δ* ^13^C_V-PDB_ and *δ*^2^H_V-SMOW_ values of synthetic reference (*E*)-cinnamic acid (1), vanillin (2), and benzoic acid (3) samples measured directly (S1) and after having been subjected to the former steps of the sample preparation procedure in the text (S1a).

Sample no	(*E*)-Cinnamic acid (1)		Vanillin (2)		Benzoic acid (3)	
	*δ * ^2^H_V-SMOW_	*δ * ^13^C_V-PDB_	*δ * ^2^H_V-SMOW_	*δ * ^13^C_V-PDB_	*δ * ^2^H_V-SMOW_	*δ * ^13^C_V-PDB_
S1	−23 ± 3	−26.9 ± 0.3	83 ± 2	−28.6 ± 0.1	70 ± 3	−28.7 ± 0.2
S1a	−24 ± 1	−26.8 ± 0.2	81 ± 4	−28.5 ± 0.2	73 ± 5	−28.8 ± 0.3

**Table 2:** Minimum (Min), maximum (Max), and average (Ave) values and standard deviation (SD) of ^2^H/^1^H and^13^C/^12^C values (‰) of (*E*)-cinnamic acid (1), vanillin (2), and benzoic acid (3) from various origins.

Origin^*∗*^	Statistical analysis	(*E*)-Cinnamic acid (1)		Vanillin (2)		Benzoic acid (3)	
		^2^H/^1^H	^13^C/^12^C	^2^H/^1^H	^13^C/^12^C	^2^H/^1^H	^13^C/^12^C
S1–S5	Min.	−42	−27.6	42	−29.0	34	−31.1
	Max.	−23	−26.9	83	−27.8	70	−28.7
	Ave.	−34 ± 4	−27.3 ± 0.3	66 ± 3	−28.6 ± 0.2	57 ± 5	−30.1 ± 0.1
N1–N4	Min.	−84	−30.7	−69	−30.6	−145	−41.6
	Max.	−63	−29.7	−28	−29.9	−128	−37.7
	Ave.	−76 ± 4	−30.3 ± 0.1	−44 ± 3	−30.2 ± 0.1	−138 ± 3	−40.1 ± 0.4
L1–L9	Min.	−103	−31.5	−82	−31.4	−156	−39.2
	Max.	−56	−29.9	−19	−29.8	−64	−35.9
	Ave.	−75 ± 5	−30.6 ± 0.3	−48 ± 4	−30.4 ± 0.3	−96 ± 5	−37.7 ± 0.4
A1		−37	−28.3	58	−24.7	40	−29.3
A2		−44	−29.5	30	−28.2	30	−33.8
A3		−61	−30.2	13	−29.6	−59	−36.3
C1		−41	−28.3	−19	−29.7	−81	−36.7
C2		−75	−30.1	−68	−30.5	−94	−37.7
C3		−44	−28.3	−18	−29.3	−90	−38.8
C4		−81	−30.3	−1	−29.2	−62	−36.9
C5		−23	−27.9	213	−26.5	−236	−38.2

^*∗*^(^■^) S-synthetic; (^●^) N-natural; (^▲^) L-laboratory prepared; (^▼^) C-commercial; (^♦^) A-adulterated. Table 2 and Figures 2–4 used the same labels.

## Data Availability

The reference data used to support the findings of this study are available from the corresponding author upon request.
